This article has been retracted.

# Blockchain-Based Trust Management Framework for Cloud Computing-Based Internet of Medical Things (IoMT): A Systematic Review

**DOI:** 10.1155/2022/9766844

**Published:** 2022-05-19

**Authors:** Mohammad Khalid Imam Rahmani, Mohammed Shuaib, Shadab Alam, Shams Tabrez Siddiqui, Sadaf Ahmad, Surbhi Bhatia, Arwa Mashat

**Affiliations:** ^1^College of Computing and Informatics, Saudi Electronic University, Riyadh, Saudi Arabia; ^2^College of Computer Science & IT, Jazan University, Jazan, Saudi Arabia; ^3^Computer Science, Aligarh Muslim University, Aligarh, India; ^4^College of Computer Sciences and Information Technology, King Faisal University, Hofuf, Saudi Arabia; ^5^King Abdulaziz University, Jeddah, Saudi Arabia

## Abstract

The internet of medical things (IoMT) is a smart medical device structure that includes apps, health services, and systems. These medical equipment and applications are linked to healthcare systems via the internet. Because IoT devices lack computational power, the collected data can be processed and analyzed in the cloud by more computationally intensive tools. Cloud computing in IoMT is also used to store IoT data as part of a collaborative effort. Cloud computing has provided new avenues for providing services to users with better user experience, scalability, and proper resource utilization compared to traditional platforms. However, these cloud platforms are susceptible to several security breaches evident from recent and past incidents. Trust management is a crucial feature required for providing secure and reliable service to users. The traditional trust management protocols in the cloud computing situation are centralized and result in single-point failure. Blockchain has emerged as the possible use case for the domain that requires trust and reliability in several aspects. Different researchers have presented various blockchain-based trust management approaches. This study reviews the trust challenges in cloud computing and analyzes how blockchain technology addresses these challenges using blockchain-based trust management frameworks. There are ten (10) solutions under two broad categories of decentralization and security. These challenges are centralization, huge overhead, trust evidence, less adaptive, and inaccuracy. This systematic review has been performed in six stages: identifying the research question, research methods, screening the related articles, abstract and keyword examination, data retrieval, and mapping processing. Atlas.ti software is used to analyze the relevant articles based on keywords. A total of 70 codes and 262 quotations are compiled, and furthermore, these quotations are categorized using manual coding. Finally, 20 solutions under two main categories of decentralization and security were retrieved. Out of these ten (10) solutions, three (03) fell in the security category, and the rest seven (07) came under the decentralization category.

## 1. Introduction

The IoMT is a rapidly expanding subset of IoT applications, in which medical devices are utilized to deliver a range of healthcare solutions. Digital technology already benefits the healthcare industry. Improved quality of life, reduced expenses, and more user knowledge can be expected from IoMT-based healthcare systems. From the standpoint of the healthcare provider, the IoMT can reduce device disruption through remote provisioning. In addition, the IoMT can accurately identify the best times to replace supplies for a number of devices to ensure their uninterrupted operation. It also allows for the efficient allocation of insufficient resources by confirming their optimal usage and the provision of new patient services through the IoMT. The IoMT devices are often worn on the body and collect various sensitive information. Caregivers and healthcare providers can use this information to make timely and data-driven decisions about an individual's health status. This information, on the other hand, is sensitive and personal. As a result, users must guarantee that their medical information is kept confidential, secure, and private. Security and privacy are two of the most pressing concerns in the internet of things. The IoMT devices are resource constrained, and they are reluctant to support the substantial resource requirements of conventional security algorithms due to resource constraints. It is also becoming more popular to develop internet-of-things (IoT) applications in a cloud computing environment since cloud computing environments have the potential to provide infrastructure and capabilities to devices that have limited resources. Because the internet-of-things devices have limited processing and storage capabilities, a cloud layer is required to complement the storage and processing requirements [1, 2]. Aside from that, the internet-of-things devices are not very safe, and the usual security strategy cannot be applied to these devices [3, 4].

The internet of medical things (IoMT) uses devices like cell phones to improve a person's health. But what makes IoMT exciting for the future is its scientific potential. Doctors and researchers can use medical gadgets to uncover new diseases and cures. For example, the public may create a global dataset documenting all individuals' clinical tales [5]. In an untrusted environment, not having a trusted context means ignoring some possible risks: personal health data are considered sensitive and should be protected. Personal and patient-centered care—IoMT—allows patients to share health data with their doctors and provide remote medical support services to maintain personal health records and manage medications. In order to address IoMT security flaws, the BCT makes use of the most recent encryption technologies.

Cloud computing has been one of the emerging research trends due to its infinite possibilities of resource sharing and enhanced user interface [6, 7]. Cloud computing is becoming a de facto requirement for providing services and scalable and efficient resources [8]. Computer services like software, databases, data analytics, servers, and networking can be delivered through the internet to provide more flexible resources, faster deployment, and cost-efficiency in terms of economies of scale. It is referred to as “cloud computing” in some circles. Cloud computing has tremendous economic importance, and it is increasingly emerging. Cloud storage services, however, actually face significant confidence and security issues. In general, the three most significant trust challenges in cloud computing are an absence of suitable information, lack of transparency, loss of control, and assurance measures. In March 2020, 5.2 million guest records were exposed due to a third-party AWS database vulnerability. Similarly, in 2019, 540 million Facebook user records and 49 million Instagram user records were compromised due to the AWS database security vulnerability of third-party applications. Also in 2019, 10.6 million user records of MGM Resorts users were breached due to cloud server vulnerability [4, 9]. In 2016, Cloudflare's platform was compromised by a flaw that leaked encrypted data from its clients, affecting at least 2 million websites [10]. For over 8 hours, Microsoft Azure's public cloud storage failures impacted similar cloud businesses. A data compromise involving Amazon Web Services resulted in the release of the U.S. voters' personal details in June 2017 [10]. A recent survey in 2020 by Check Point Inc. highlights that 82% of users feel that traditional security strategies cannot handle the cloud security threats, and 52% consider that the public cloud is more vulnerable than the conventional environment [11]. All these issues and surveys point to the lack of user trust in the cloud environment and inherent problems of trust management even after a lot of development in the field of cloud computing.

Many scholars have reviewed the aspects of trust management in cloud computing. Li et al. have implemented a novel approach to trust that allows cognitive behavior to be analyzed and predicted by users [12, 13]. Trust models, together with evolutionary algorithms, have also been introduced [14, 15], as have many useful techniques for trust-enabled service management [16, 17]. However, the conventional trust paradigm typically depends on a centralized trust control center for third parties, leading to delays, congestion, and possible single point of failure. Furthermore, in a centralized trust system, as proof of trust is not revealed to all users, the findings of the trust assessment are entirely verifiable by the users. Medical data can be stored and processed in the cloud using IoMT devices connected to cloud services. Cloud-based IoMT security, privacy, and trust issues rapidly arise. Researchers recently paid increased attention to security, privacy, and trust [2]. Data security ensures the data's integrity, validity, and, most crucially, authenticity. It also ensures that only authorized individuals can read and modify data. Privacy preservation is another important goal to keep in mind when constructing IoMT. It accounts for the severity and sensitivity of materials shared across an open and insecure channel. Privacy preservation involves content and context. Content privacy protects patient data from leakage, but patient privacy is difficult to achieve because an attacker can identify patient health based on the attending doctor's identity. Contextual privacy is also critical. Protecting the communication's context is a contextual privacy. Various symmetric and asymmetric encryption methods are utilized in IoMT-enabled healthcare systems. Recent research shows that using advanced machine learning (ML) techniques on resource-constrained devices like IoMT is not optimum. The solution is to use simple privacy-preserving methods on IoT devices and the cloud for complicated ML algorithms. Many studies have been published on cloud-based IoMT security in healthcare systems.

Blockchain technology has gained recognition and usage in cryptocurrency, security, trust management, and immutability features. In the absence of a third party, the system's robustness is unaffected by the failure of a few nodes. Transparency, nonrepudiation, and confidentiality are all ensured by the use of digital signatures and the data chain and consensus processes in the operational rules and data documents. When it comes to the creation of a modern decentralized trust model, the decentralization aspect of the blockchain is very important [18]. Blockchain offers a modern way to create a trust-enabled cloud computing environment [19, 20]. Blockchain can also be a possible solution in this environment to provide security, trust, and authentication services. To date, a number of researchers have proposed a blockchain-based solution for trust management, which has garnered widespread attention. In this study, we have examined a variety of pertinent topics and examined, classified, and contrasted them. On the other hand, blockchain-based trust building in a cloud-based system is fraught with problems and difficulties, such as blockchain assaults, the high overhead of consensus mechanisms, and delays in real-time transaction processing. Furthermore, this work provides various suggestions for future research in the area of blockchain-based trust management.

The following are the most significant contributions made by this study:

  The existing blockchain-based trust techniques are reviewed for cloud computing systems.
  On the basis of established parameters, the various blockchain-based trust techniques are compared for cloud-based systems that were accessible.
  Cloud computing and IoMT and their layered architecture are integrated.
  Prospective research directions are identified in blockchain-based trust management for cloud-based systems.
  Research is suggested for future work, i.e., integrating IoMT with blockchain and machine learning, 6G, and the effect of quantum computing on IoMT.

## 2. Background Study

This section discusses the primitives like trust in cloud computing, the challenges of trust management, and the basics of blockchain.  Table 1 reviews the related literature surveys on trust approaches using cloud computing and blockchain technology.

### 2.1. IoMT and Cloud Computing

An IoMT platform is a smart structure that essentially encompasses sensors and electrical circuits for the acquisition of biomedical signs from a patient and a processing unit for the processing of biomedical signs. Additionally, it includes a network device for data transmission across a network, a storage unit, and a visualization platform for making judgments based on the ease of medical practitioners. It enables the physician to perform routine activities, while patients are continuously monitored and benefit from the home setting. Traditional remote monitoring systems are inconvenient for patients due to the size of the components involved in the body and the requirement for regular charging or changing of batteries. The IoMT revolution tackles the aforementioned challenges by designing compact, ultra-low power sensors and lightweight communication procedures.

It is expected that IoMT-based healthcare systems will improve users' quality of life, cut expenditures, and expand their knowledge. The IoMT can reduce device interruptions through remote provisioning from a provider healthcare standpoint. Additionally, the IoMT can accurately determine the optimal times to replace supplies for several devices to ensure their continued and smooth operation. Additionally, the IoMT enables appropriate scheduling of scarce resources by confirming their optimal utilization and service to new patients. The primary issues associated with IoMT applications are similar to those associated with IoT. They center mostly around user privacy, authentication, data security, integration with heterogeneous devices, and the resource-constrained nature of devices. Cloud computing is a technology that enables the provision of massive amounts of resources and computer services across a networked platform, such as the web. In its simplest form, cloud computing brings up the use of servers connected to the internet for the storage, management, and processing of data. It benefits potential users by enabling them to access virtual hardware, collaborative software, and virtual storage and servers.

Cloud computing uses the internet to provide computer services such as databases, servers, software, data analytics, and networking to give flexible resources, rapid response, and scalability. The IoMT devices can communicate with medical data storage and processing systems that are hosted in the cloud. Cloud computing and IoMT are generally integrated into three-layer architecture that is been shown in Figure 1. These three layers are (1) the IoMT layer, (2) the fog layer, and (3) the cloud layer. The IoMT devices that include sensors, actuators, and other medical devices for monitoring are all included in the IoMT layer. The layer directly works with the patients and other healthcare system users. This layer collects data from patients. Between the cloud and the object layer is the fog layer. This layer is composed of local servers and gateway devices that provide the foundation of a sparsely distributed fog networking infrastructure. The devices at the lowest layer use the local processing power to provide real-time responses to their consumers.

Additionally, these servers are utilized to oversee and administrate the system's security and integrity. This layer's gateway devices are in charge of forwarding collected information to the upper layer and act as middleware. The storage and processing of these forwarded records are performed at the cloud layer and based on this analysis; the decisions are made. It will store data generated by the medical infrastructure and undertake analytical work as needed in the future.

### 2.2. Research on Trust Issues in Cloud Computing Systems

Trust management offers a creative approach to addressing security issues in heterogeneous, transparent, distributed, and rapidly evolving networks [32–36]. Trust includes the features of subjectivity, fuzziness, ambiguity, context asymmetric, and minimal transitivity. Trust can be classified into four categories depending on various classification approaches [37].

  Unified, direct, and indirect trust: it is based on the recommendation and the trust acquisition approach used.
  Behavioral and identification trust: trust is based on identification.
  Function and expertise trust: it is based on the timing and occurrence of trust.
  Objective and unobjective trust: it is based on the representation of trust.
  Internal domain and cross-domain trust: it focuses on trust groups.

A trust model is a model that models, measures, and tracks a confidence connection. The trust model can be divided into centralized and decentralized models based on the trust management model. The principal trust server is accountable for storing, updating, and maintaining both stakeholders' trust data for the centralized trust architecture, which must be completely correct and uncompromising. Furthermore, utilizing a centralized trust model will result in significant latency and a single point of failure, lowering the quality of cloud services (QoS). Some researchers consequently suggested a decentralized trust model. For instance, EigenTrust [38] and PeerTrust [37] are the popular decentralized trust models.

### 2.3. Trust Approaches and Challenges in Cloud Computing Systems

At present, cloud researchers focusing on trust-based methods face significant theoretical and implementation challenges. Some of these are as follows:

  Several trust models are centralized: many of these pretend to be decentralized models that also require a third-party trust center or maybe even validation center, which results in security risks including a single point of failure, overload and loss of credibility, etc.
  Proof of trust is not available to all cloud participants and cannot be traceable; hence, the findings of the trust evaluation were not entirely trusted by each individual.
  The inconsistency for the result of trust evaluation: current trust models lack adequate definition capability (a data type is comparatively fundamental and often in numerical scores) and are incompatible with actual implementations like e-commerce input from people requiring multiple data types.
  Less adaptable: subjective approaches are used in trust decision-making. Subjective methods make the model subjective, lacking in empirical and adaptability. Different subjective methods include expert scoring and averaging process. The trust model is inaccurate for malicious attacks.
  Enormous overhead management results in several pitfalls and shortcomings in practical implementation; thus, it was inappropriate for large communication networks.
  Many trust models perform performance tests through modeling trials, which need further assessment.

#### 2.3.1. Blockchain Technology

In 2008, Nakamoto first proposed the idea of blockchain called Bitcoin Framework. This study further explains the full notion and technological details of the arbitrator-free payment scheme aiding entities to make and accept disbursements without needing a financial intermediary [39–41]. Broadly, it is categorized as a distributed ledger that is cryptographically encrypted to be untampered and unforgettable. Blockchain is a distributed architecture containing a cryptographic standard that provides a particular data structure for data authentication and storage and a distributed consensus framework for data creation. Cryptographic methods for information security and smart contracts are used for automated data analysis and actions [42].

There usually exist three blockchain forms: public blockchain, private blockchain, and hybrid blockchain. The blockchain's main characteristics are to provide the following: decentralization (did not depend on middleware and did not have central control), open source (open-source data and open public interface), autonomy (based on consensus processes and dynamically and securely operating in the absence of human intervention), and secure (data are secure and tamper proof as per regulations and policies) [43, 44].

#### 2.3.2. Blockchain Architecture

Blockchain largely depends on peer-to-peer networks, asymmetric encryption algorithms, blockchain, and digital currency. Blockchain consists of three layers: infrastructure, technical, and support. The infrastructure layer has two semilayers: (1) network and networking layer, and (2) data layer. The semilayer network and communication include decentralized peer-to-peer technology, multicast technology, and networking and blockchain experiences. The data semilayer primarily contains the distributed storage architecture and file system implementing the blockchain data structure and developing, testing, and maintaining blockchain data [45]. The technological support layer offers technological backing to the blockchain. The technology support level comprises the elements needed to integrate blockchain deployment and participation control [46].

## 3. Blockchain Technology for Trust Management

Blockchain has demonstrated its utility as a decentralized database that anybody may access. Composing or upgrading in such a repository occurs in an open, secure, and decentralized manner, allowing all readers to see the same prewritten values. Although it is commonly used for financial services and cryptocurrencies, identity authentication and access control for cloud/IoT have been recently investigated as another possible application of technology [47]. Identity authentication assures cloud market participants, including customers and service providers. Usually, the third-party management center requires a conventional identity management approach. The authentication center provides services of identity authentication on request to cloud entities. It can effortlessly lead to security threats and risks, such as excessive certification center authority and single point failure. Identity federations are one of the alternative solutions that are broadly distributed systems to address security and trust problems across multiple domains, though they increase system design and operational complexity [48]. Weak trust management brings many issues of stability, privacy, security, and interoperability to cloud computing. Therefore, in conjunction with blockchain technology, there is a need to design a decentralized trust system.

## 4. Research Methodology

### 4.1. Systematic Review Execution

This systematic review involves six phases, i.e., (1) identifying the investigation question, (2) research methods, (3) screening of the related articles, (4) abstract and keyword examination, (5) data retrieval, and (6) mapping processing.

### 4.2. Research Question

Prior knowledge of research questions is vital in advance of the research being conducted. These are the research questions related to the challenges of trust in cloud computing and the effect of integration in IoMT.

What are the challenges of trust in the cloud computing environment?

The research question is critical for identifying different trust challenges in cloud computing environments. In particular, it is essential to review the related articles in scientific databases to recognize the unique trust challenges that require solutions. Then, the map of the trust challenges can be presented after the challenges have been classified.

Which blockchain-based approaches/solutions are available for the identified challenges in the cloud computing environment?

Despite the many approaches/solutions suggested to solve the identified challenges, not all have been successfully implemented. Numerous challenges can be established in real-world implementation by reviewing the related papers. Thus, it is vital to consider mapping the solutions to the challenges. These solutions will illustrate the research gap and guide future research.

How are the challenges currently being addressed?

This research inquiry targets to understand the blockchain-based trust management suggested by researchers as a reference for forthcoming projects. These applications and resolutions must be categorized according to mapping methods. Notably, numerous changes and enhancements were made. As a result, clear guidelines could be made on promising investigation scenarios for blockchain-based approaches for managing trust in cloud computing.

## 5. Conducting Research

Various approaches are required for conducting this research, including searching strategy, and criteria for inclusion and exclusion for coming up with a substantial outcome discussed in this section.

### 5.1. Information Sources and Search Process

The research was first performed using the keyword approach to retrieve related articles. To look for academic articles and abstracts, the keywords searched are “trust,” “blockchain,” and “cloud computing.” A systematic search was performed on scholarly databases like IEEE Xplore, Scopus, the Web of Science, and the ACM Digital Library. Subsequently, all the selected papers are downloaded from the earliest to the latest publication. We adopted the PRISMA guidelines, as shown in Figure 2. Apart from searching for the databases, reference lists of the downloaded articles were manually scanned to find any other related research that would be included in the study. In this phase, a total of 319 articles are obtained.

### 5.2. Inclusion/Exclusion Criteria

When the questions regarding the scope were identified, all research articles were considered to determine relevant details for the systematic analysis of this research. The selection of the article was performed based on a collection of criteria for exclusion and inclusion (see Table 2) for the study of highly significant literature.

The abstracts of all research works were initially reviewed. Articles satisfying one of the criteria for exclusion are excluded. In this case, 151 papers were omitted as they evidently focused on “trust” rather than “trust in cloud computing”; moreover, 64 articles were excluded because they clearly focused on blockchain and cloud computing rather than “blockchain,” “trust,” and “cloud computing.” Then, the remaining 104 articles are inserted into the Mendeley software to remove the duplication and merging of articles, resulting in a reduction of 13 articles.

### 5.3. Searching Process

To precisely match research questions with the content of the chosen papers, we have read a full text and conducted a process to make the paper selection finer. Also, we examine the title and abstract of each selected article. The contents of abstracts that concentrate less on main topics or with less specific findings to the group of information have been excluded to ensure consistency and academic standards. We have removed 57 articles because they are less relevant to our scope of the research. In this last stage, 34 articles were obtained for this analysis. Figure 2 demonstrates the technical steps for paper assortment and provides assortment criteria or major filter actions for the most related articles.

### 5.4. Screening Process

Each article generally presents essential keywords after the abstract section. From the finally selected paper for quantitative analysis, 34 keywords were obtained after entering them into quantitative analysis software (Atlas.ti). The keywords for this systematic review were “trust,” “blockchain,” and “cloud computing.”

### 5.5. Data Abstraction and Mapping Process

The selected keywords were used with Atlas.ti software to search for related articles. It led to the collection of about 70 codes and 262 quotations from the analysis. The codes were then manually coded to identify the quotes. However, the codes were conducted into the network for the mapping process. Finally, the relation between the codes is created in the network, which is shown in Figure 3.

## 6. Results

The result of a systematic review is given in this section. A total of 319 papers are accumulated from different databases. We excluded the 151 articles in the first screening as they clearly focus on trust rather than trust in cloud computing. Additionally, 64 articles were omitted as they focus on applying blockchain in cloud computing rather than blockchain, trust, and cloud computing. Then, the remaining 104 articles are inserted into the Mendeley software to remove the duplication and merging of articles, resulting in a reduction of 13 articles. In the next phase, the full text of the article is screened based on defined criteria for finer selection, resulting in a reduction of 57 articles because they are less relevant to our scope of the research. Finally, 34 articles were obtained, which is the basis for our study and added to the reference section of this research study.

## 7. Discussions

Currently, research on cloud computing trust approaches faces enormous theoretical and implementation challenges.  Table 3 provides a comparison of trust-based approaches in the cloud computing environment.

## 8. Additional Points of Trust Challenges in Cloud Computing

### 8.1. Centralized

Owing to the lack of centralized trust management, an independent quality assurance entity should be charged with ensuring customer trust information based on knowledge when choosing cloud providers. Many trust models were centralized, and most of those claiming to be decentralized models often needed a third-party trust center or a certificate center. This results in several security challenges, such as a single failure point, overload, and center node's reputation [51, 54, 55, 57–59].

### 8.2. Trust Evidence

Cloud center data are stored at various locations at varying virtualization speeds. Present leading CSPs (e.g., Microsoft Azure and Amazon EC2/S3) do not have full physical and virtual server transparency [60]. Customers now only have the transparency to view virtual machine performance metrics and track event logs. Enhanced transparency would improve customer trust in the cloud. Trust evidence does not apply to all cloud organizations and cannot be tracked, so the outcome of trust assessments is not reasonable or not trusted by all participants [53, 55, 58].

### 8.3. Inaccuracy

The trust feedback for the reliability of the user is difficult to obtain. Malicious users may intentionally distribute mistrust information to damage the credibility or falsely increase some nodes' credibility. The involvement of an independent quality assurance body to provide consumer trust may solve the problem of assessing the credibility of the trust feedback and the inaccuracy of the trust assessment findings. The traditional trust models lack adequate definition and are inaccurate with actual applications. The type of data is extremely straightforward and is mainly in number form, like e-commerce, for which input of individuals always requires different kinds of data such as numerical and character [52, 53, 56].

### 8.4. Less Adaptive

The trust evaluation method makes use of subjective approaches such as expert grading and averaging, which results in subjective, scientifically ineffectual, and adaptive trust models. Trust models were insufficiently resilient to deal with malicious (collusion) attacks, particularly those involving malicious behavior [49, 50, 54, 56, 59].

### 8.5. Huge Management Overhead

Mostly in cloud computing platforms, one job can be spread over many computer nodes. Multiple tasks can share a single compute node. In such instances, tasks may be shared with other untrustworthy tasks or environments. When involving multiple cloud systems, consideration should be given to load balancing and redundancy and the trustworthiness of computer nodes, node groups, tasks, or cloud computing environment. Huge overhead management leads to several shortcomings in the real implementation, like approaches in large-scale multiple cloud systems such as distributed data sharing and remote computing that are not acceptable [49, 50, 52, 53, 57].

## 9. Summary of Blockchain-Based Trust Solution in Cloud Computing

Table 4 provides the solutions categorized into two major areas of decentralization and security for cloud computing based on the review of the related research articles. Figure 3 demonstrates the trust solutions and problems mapped using Atlas.ti version 8.0 to present the mind map of categorization. It is followed by the particulars of the results discussed in the section on decentralization and security.

### 9.1. Decentralization

In [61], it has proposed a new cloud data sharing architecture based on blockchain technology to enable equitable data distribution and data protection in a multicloud environment. The architecture was divided into four components: the blockchain network, cloud customers/users, data owners, and data service agents (a third-party agency). After establishing their identity and evaluating blockchain authorization, users submitted data sharing requests via the service agent and were provided with the relevant data service. The suggested approach employs a Shapley value-based incentive mechanism that is further validated using the SVM model and generates mining revenue via PoW, PoS, and PEFT consensus mechanisms. Zhu et al. (2019) designed a controllable blockchain data management (CBDM) model for cloud computing [62]. It used both the normal voting nodes and the third-party higher-level trust authorities for transaction verification. The model provides data management in a controlled manner and increases efficiency and trust. It utilizes a SaaS service for cloud storage. This scheme proposes two new user registration and voting and counting algorithms. A key generation scheme based on bilinear pairing techniques has been used to provide security to the system during the registration process. Access control is a methodology to restrict access or control access to protect the corporate and user's personal data in the cloud. However, centralized access management techniques frequently result in the loss of data integrity, privacy leaks, and the possibility of hacker assaults. To address these challenges, a blockchain-based access control architecture-dubbed AuthPrivacyChain has been suggested and deployed based on enterprise operations [63].

The AuthPrivacyChain designed an access control and identity authentication mechanism to address the entities in the blockchain with unique IDs. Using blockchain's decentralized nature, the distributed and decentralized control system for cloud access has been introduced, thereby improving the privacy and security of data applications. The proposed model provides access control in the form of decentralized access control, revocation using revocation authorization, and privacy protection using the AES encryption algorithm. It refines users' data protection and privacy and effectively resists internal and external attacks. Cloud computing has become a vital technology in the era of industry 4.0 for globalization and intelligent computing development. Cloud manufacturing faces many technological challenges—including security, reliability, data manipulation, and single failure points, constrained by conventional centralized architecture and third-party trust entities [64].

The paper [65] applied a collaboration arrangement between consumers and resource providers using the blockchain-based decentralized cloud manufacturing application model. A smart contract named blockchain-based DCMApp (decentralized cloud manufacturer application) was used for the provision of service under the agreement. It uses an IPFS for storage and anyone from PoS, PoW, or DPoS for a consensus mechanism. The cloud service-level agreement (SLA) does not always assure that it can be credibly implemented and automatically as expected. This study introduced a conventional SLA service model and named it witnesses, containing cloud service interaction protocol [61].

The role is to detect service infringements and guarantee the credibility of data transactions. The proposed model obtained benefits from cloud transactions in which the witnesses are the ordinary nodes of the blockchain network. The witness model basically comprises three attributes: witness selection, violation detection, and audit. Witness selection uses the Nash equilibrium principle; the audit mechanism uses the payoff function and violation detection through the unbiased sorting algorithm. Witnesses assist by monitoring the transactions to successfully proceed and oblige all parties to fulfill their credit obligations. In conventional cloud storage for data deletion, the single-bit return protocol is typically used, which can easily result in unreliable deletion. However, some deletion strategies have drawbacks, such as nonverifiable deletion results requiring third-party trust for confirmation and low-efficacy tests.

A blockchain-based data deletion framework was implemented by [62] to boost verification, reliability, efficiency, accountability, and transparency. The proposed secure data deletion scheme has two main functionalities: transparency and malicious behavior detection. A publicly verifiable data deletion scheme provides transparency, and cryptographic primitives such as ECDA along with timestamping provide malicious behavior detection. Both file/data operations are registered in the blockchain to guarantee the data deletion on the server is truthful. K. Bendiab et al. (2018) proposed a novel blockchain-based identity management model, which accords the operative trust authority service to cloud computing schemes [63]. This model permits the service vendors to establish the relationship of trust behavior with the customers and other stakeholders in a distributed, dynamic, and decentralized manner without the central authority's interference. The model covered three significant trust factors: authentication, user integrity/creditability, and satisfaction, to be described and computed. It uses user feedback for credibility, user anomaly detection for authentication, and satisfaction to evaluate user satisfaction.

### 9.2. Security

This study proposes a blockchain and SDN (software-defined networking)-based hybrid cloud service architecture to resolve the security issues associated with conventional centralized cloud architectures [67]. It enhances the integrity using the MD5 hash algorithm and identifies malicious hosts using the IP-MAC address. It further enhances the availability of cloud platforms using autonomous bandwidth provisioning. The proposed architecture had two major parts—the multicontroller SDN network layer and a blockchain security management layer.

The architecture included a sublayer for edge computing and for P2P (peer-to-peer) network routing. The author presented a novel model that utterly tracks and validates the cloud commands, detects malicious nodes, and upsurges the availability and accessibility of cloud services. J. Li et al. (2018) proposed a distributed blockchain-based cloud storage security architecture. They customized a genetic algorithm to enhance storage performance and security by solving the replica distribution problem [69]. The suggested architecture divides user files into equal-length file blocks and stores them in the P2P network, encrypted and digitally signed. Blockchain-based transactions were meticulously documented in each secure block's body, which is traceably organized.

Generic algorithms are used to resolve the issue of copy replacement between multiple centers and users. It further utilizes the ECDSA encryption algorithm for file security and uses the Merkle Hash tree with SHA-256 algorithms for file verification. It additionally uses a genetic algorithm-based data redundancy scheme for fault-tolerant file storage. Paper [71] proposed a precise Ethereum public blockchain-based timestamping scheme called Chronos + for data outsourcing. In Chronos+, cloud service providers offered both storage and timestamp services to ensure accurate, reliable, efficient, secure, and scalable file storage services. This scheme utilizes the AES algorithm for security and supports batch timestamping for better efficiency. It further includes orthogonal schemes for providing integrity of records.

## 10. Future Research Work

Various aspects of trust issues in cloud computing and IoMT have been discussed in the discussion section. Still, some areas of concern need to be further researched for the efficient and trustful application of cloud computing-based IoMT. These aspects have been summarized in this section.

### 10.1. Malware and Intrusion Detection

Malware and intrusion are the most probable security attacks on IoT systems and that also apply to IoMT. These aspects were not researched a lot in the beginning, but now it becomes imperative due to the involved life risks and reliability of devices. Machine learning-based approaches are being actively used for malware and intrusion detection in IoT devices. Still, due to memory and processing constrained, an efficient approach and algorithm are required for successful implementation [72].

### 10.2. Energy Efficiency Solutions

The IoMT sensors and devices are resource-constrained devices with limited capacity that need to securely and reliably communicate for critical healthcare solutions. Failure of any such device will be life-threatening; therefore, power consumption efficiency is more critical for these applications for long-term hassle-free applications. Energy-efficient routing protocols are also very important for resolving the energy efficiency issues in IoMT and the long-term use of such devices without any interference.

### 10.3. Integration with 6G

Although the 5G network has been available for a while, various research studies have been performed on the 5G integration with IoT networks. However, 6G is still a new phenomenon, and its integration with IoMT needs to be thoroughly investigated, and related use cases need to evolve for its integration in healthcare applications [73].

### 10.4. Integrating Edge Computing, Machine Learning, and Blockchain

Various efforts are going on to integrate edge computing, machine learning, and blockchain with IoMT to provide a safe, reliable, and efficient approach for healthcare applications. Many kinds of research studies have been performed in the recent past, but still, many opportunities are available to integrate them into various aspects of healthcare and medicine development [74].

### 10.5. Quantum Computing and Effect on IoMT

The threats from the quantum computing evolution are evident due to the high capabilities for processing instructions. The traditional encryption approaches will be toothless in providing security in such an environment. Although several approaches are available for secure quantum algorithms, these cannot be suitable for resource-constrained IoMT devices. These aspects need to be evaluated and researched further on [75].

## 11. Conclusions

This study has reviewed the existing literature on trust management approaches for cloud computing. It has provided challenges of trust issues in a cloud environment and possible use cases of blockchain adoption. The challenges of cloud computing compiled in this study are centralized, huge overhead, trust evidence, less adaptive, and inaccuracy. Blockchain-based trust approaches are been given in Table 5 based on function, application scenario, and blockchain type used and also describe the focus/contribution. Furthermore, solutions to these challenges based on the category and application domain of solutions are given in Table 6, which have been further categorized into two main areas: decentralization and security. Three (3) fell in the security category out of these ten solutions, and the rest of seven (7) came under the decentralization category. This study shows the security and centralization challenges and then their solutions in the form of a mapping tree. These solutions highlight the role of blockchain technology in managing trust in cloud systems and cloud-based IoMT and further provide future research topics for research in this domain.

## Figures and Tables

**Figure 1:** Architecture of IoMT and cloud integration.

**Figure 2:** PRISMA flowchart.

**Figure 3:** Mapping of trust challenges with the solution.

**Table 1:** Review of related literature surveys on trust approaches.

Ref	Idea of paper	Year	Blockchain	Cloud	Trust
[21]	Overview of customer trust in cloud computing schemes to improve service provider behaviors	2016	x		
[22]	Review of trust approaches in cloud systems	2016	x		
[23]	Analyze the trust models in cloud systems	2018	x		
[24]	Overview of attacks and existing trust techniques in cloud system	2017	x		
[21]	Survey of trust in the cloud computing system	2016	x		
[25]	Analysis of evaluation methods for trust in cloud computing systems	2018	x		
[26]	Review of trust models and evaluation methods for a cloud system	2016	x		
[27]	Survey of trust evaluation methods and factors for cloud computing systems	2017	x		
[28]	Use of blockchain for making a trust-free system	2020		x	
[29]	Review application of blockchain in IoT cloud-based systems	2019			x
[30]	Discuss the blockchain infrastructure for cloud and performance comparison of cloud data center	2020			x
[31]	Review of attacks on blockchain and existing solutions	2019		x	x
This study	Blockchain application for trust management in cloud computing based IoMT	2022			

**Table 2:** Inclusion and exclusion criteria.

Selection criteria	Details
Exclusion	(i) Non-English journal
	(ii) Published between 2015 and 2021
	(iii) Duplication
	(iv) Title and abstract not related to the scope of the paper

Inclusion	(i) Title and abstract related to trust in cloud computing
	(ii) The given solution must be evaluated

**Table 3:** Comparison of trust-based approaches in cloud computing.

Ref	Focus	Strengths	Type	Software used	1	2	3	4	5
[49]	Provide a trusted service brokering scheme to deal with multiple user requests for cloud resources	Robust in managing different dynamic service behavior at numerous cloud sites	Prototype	Eucalyptus—cloud environment				Y	Y
[50]	Provided a trust evolution approach for cloud computing to eliminate the limitation of the existing trust model	It includes factors like user requirements, aggregates qualitative and quantitative evaluation, and incorporates user feedback in the trusted computing	Trust evaluation approach	--				Y	Y
[51]	Proposed a trust model for a cloud application to address the security issues	1. Trust function in the given trust model to secure from a security attack	Model		Y				
		2. The developed trust model provides integrity, access control, availability, and privacy							
[52]	A fuzzy logic-based trust calculation scheme by which trust is provided by service provided to the participants	To determine the trustworthiness of the cloud supplied using a fuzzy logic-based rating approach to convert the result and compliance values into rating	Scheme	MATLAB			Y		Y
[53]	A trust evaluation model based on fuzzy logic to predict trust values	Prediction of trust value based on clouds' user feedback	Evaluation model	MATLAB		Y	Y		Y
[54]	An SLA-based trust model was developed using user behaviour evaluation	Selection of cloud provided based on the SLA parameters	Model	MATLAB	Y			Y	
[55]	A trust model in insecure clouds based on domain partitions to address the issue of overhead and performance of cloud system	Efficient and accurate computation of trust	Model	MATLAB	Y	Y			
[56]	A trust management framework for securing the platforms of cloud computing	Allows the administrator to make decisions and manage the degree of redundancy and cost of resources	Framework	---			Y	Y	
[57]	A trust architecture allows cloud customers to make decisions about cloud providers based on their reputation	Low overhead	Architecture	N/W simulator	Y				Y
[58]	A trust management system to evaluate trust and reputation	The system developed is secured and maintains the trust and reputation of the cloud service provider	Evaluation management system	--	Y	Y			
[59]	A trust evaluation model for improving trust	Robust and secure	Evaluation model	MyEclipse	Y			Y	
Challenges—1. Centralization. 2. Trust evidence. 3. Less adaptive. 4. Huge management overhead. 5. Inaccuracy.									

**Table 4:** Category of solutions.

Challenges	Solution
Centralized	Decentralization
Huge overhead	
Trust evidence	
Less adaptive	
Inaccuracy	Security

**Table 5:** Summary of blockchain-based trust approaches.

Ref	Publish year	Function and application scenario	Blockchain type	Focus/contribution
[66]	2020	Access control framework	Public blockchain	Developed a decentralized identity management system
[61]	2019	Cloud service transactions	Ethereum	Proposed a conventional SLA service model to detect the service infringements
[67]	2020	Cloud security architecture	Ethereum	Proposed a blockchain and SDN-based hybrid cloud service architecture for cloud security
[65]	2020	Cloud manufacturing	Ethereum	A new blockchain-based cloud manufacturing application model for interaction agreement
[68]	2020	Data sharing in multicloud	Consortium blockchain	Architecture for equal data distribution in a multicloud setting in a secure manner
[62]	2018	Data deletion in cloud storage	Public blockchain	Proposed a blockchain-based data deletion scheme to boost verification, reliability, efficiency, accountability, and transparency
[63]	2018	Cloud identity management	Public blockchain	Provide a model to manage trusted behaviors and relationships with users without a centralized authority
[69]	2018	Cloud storage based on P2P architecture	Not clear	A blockchain-based framework to counter data security, single point of failure, and privacy leakage issues in file block replica placement using genetic algorithm
[70]	2018	Cloud data management	Ethereum blockchain	Proposed a controlled cloud data management model to counter lack of control and other potential security threats
[71]	2020	Blockchain timestamping scheme	Public blockchain	Proposed a blockchain-based time stamping scheme to ensure accurate, reliable, efficient, secure, and scalable file storage services

**Table 6:** Solutions for trust issues.

Ref	Solutions	Category	
[68]	Secure and collaborative data sharing	Data sharing	Decentralization
[70]	CBDM: cloud data management	Data sharing	
[66]	AuthPrivacyChain	Access control	
[65]	BC-DCM app	Access control	
[61]	Witness model	Trust model	
[62]	BC—data deletion scheme	Trust model	
[63]	WIP: blockchain trust model	Trust model	
[67]	BC-SDN	Security	Security
[69]	Blockchain-based security architecture	Security	
[71]	Chronos: blockchain-based timestamping scheme	Security	

## Data Availability

It is a review article, and no data were used to support this study.
